# Technology Acceptance in Socially Assistive Robots: Scoping Review of Models, Measurement, and Influencing Factors

**DOI:** 10.1155/2022/6334732

**Published:** 2022-07-22

**Authors:** Ying He, Qiu He, Qian Liu

**Affiliations:** School of Medicine, Hunan Normal University School of Medicine, Changsha, Hunan, China

## Abstract

**Objectives:**

We summarized technology acceptance and the influencing factors of elderly people toward socially assistive robots (SARs).

**Methods:**

A scoping review whereby a literature search was conducted in Embase, Cochrane, Scopus, PubMed, and Web of Science databases (2006–2021) to retrieve studies. No restrictions on study methodology were imposed.

**Results:**

Out of the 1187 retrieved papers, 35 studies were finally included in the study. The articles covered various aspects, including general attitudes towards using SARs, technology acceptance theory models, and factors associated with technology acceptance. Twelve studies reported a positive attitude towards SARs. Three explicit theoretical frameworks were reported. Studies involving the elderly reported three themes that influence attitudes towards SARs: individual characteristics, concerns/problems regarding robots, and social factors.

**Conclusions:**

This review elucidates on the suitability of theory-based framework as applied to acceptance of SARs. We found that research on technology acceptance with regard to SARs is still in the developmental stages, and further studies of assessment tools for SARs are required. It is also essential to consider the factors that influence the acceptance of SARs by older people to ensure that they meet the end goal requirements of the user.

## 1. Introduction

Due to improving human life expectancy, the increase in the global elderly population exhibits a continuous and steady growth trend [1]. It is predicted that by 2050, there will be more than 2 billion people aged over 60 years in the world, and that the proportion of the elderly population will be one-fifth of the global population [2]. The rapid growth of the elderly population is associated with severe health and economic challenges, coupled with shortage of nursing resources. Therefore, there is a need to establish approaches for ensuring the quality of life and medical care of the elderly [3].

Socially assistive robots (SARs) were defined in 2005 as a technology that establishes close and effective interactions with users to provide help and support in rehabilitation, companionship, and safety among others [4]. It is an invention that can effectively alleviate the challenge associated with elderly care. SARs are mainly classified into service robots and companion robots [5, 6]. This technology can help the elderly implement cleaning, cooking, medication reminders, shopping, safety reminders, and health monitoring and provide online video communication [2]. Thus, it plays an essential social promoting role in the life of the elderly by improving the independent living ability as well as the connection between the elderly and the outside world. Improving the physical and mental conditions of the elderly through SARs can reduce caregivers' burden and save medical resources.

An increasing number of studies have focused on technology acceptance of SARs [5, 7]. This is because the significance of SARs can only be realized if people accept, embrace, and use this technology. Ezer et al. reported that older people generally have positive attitudes towards robots, and they are more willing to use robots to complete tasks [8]. With regard to factors that affect the use of SARs by the elderly, Broadbent et al. reported that the types and functions of SARs and various contextual factors, including personal and robotic, influence the acceptance of SARs [2]. Technology acceptance is a significant challenge faced by designers and users of SARs. Various technology adoption models have been proposed to explain user adoption of new technologies and to assess the factors that affect user acceptance. They include Technology Acceptance Model (TAM) [9], Unified Theory of Acceptance and Use of Technology Model (UTAUT) [10], and Almere Model [11]. TAM suggests that attitudes have a direct effect on willingness to use. UTAUT states that user behavior intentions and use behavior of information systems are mainly affected by four factors: performance expectations, effort expectations, social influence, and convenience conditions. In Chen's research, performance expectations, effort expectations, social influences, convenience conditions, and hedonic expectations were shown to positively affect user adoption of escort robots, resulting in usage behaviors [12].

However, in the past few years, there have been significant changes in terms of instrumental and social abilities of SARs. For example, the elderly gained emotional interactions through chatting, entertainment, and mutual improvement with SARs [13]. It is suggested that robots are becoming more functional and focusing more on emotional interactions [14]. These functional changes bring new challenges that affect technology acceptance. Wu et al. showed that older adults remain technologically uneasy, feel stigmatized, or are confused about ethical/social issues related to the use of SARs [15]. In general, acceptance of SARs among the elderly is affected by various factors [16]. However, a limited number of review articles have comprehensively summarized previous studies on technology acceptance models, measurement, and influencing factors of SARs.

This review summarizes the results of previous studies on socially assistive robots in elderly care, including analyses on acceptance and influencing factors for the use of social assistance robots. Our findings inform on the development of future robots.

## 2. Methods

### 2.1. Study Design

A scoping review was performed to map relevant literature in the field of SARs. In contrast to systematic and narrative reviews, scoping reviews focus on an initial appraisal of current extent, scope, and nature of research literature. Furthermore, the method tends to address broader problems where many different study designs may be applicable. It is also considered appropriate because it takes the dissemination process one step by summarizing the relevant research activities in existing literature. Using the framework developed by Arksey and O'Malley [17], we examined a range of theory models, measurements, and impact factors of technology acceptance, and no restrictions on study methodology were imposed.

### 2.2. Search Strategy

Five databases, including Cochrane, Embase, PubMed, Scopus, and Web of Science, were searched to find relevant articles for the present review. The selected articles were on attitudes of the elderly towards SARs, factors affecting the acceptance of SARs and had only been published between October 2006 and September 2021. The main search was conducted on April 2, 2020, and the latest search was conducted on September 30, 2021.

The database search query was composed of three search concepts: participants (the elderly), the intervention (socially assistive robots), and the outcome (acceptance). Free-text terms for participants included “aged,” “aging,” “elder∗,” “senior∗,” “adult∗ user∗,” “older person∗,” “old people,” “older people,” and “old∗ adult∗”; their associated MeSH term was “Aged, 60 and over.” Free-text terms for the intervention included “service robot∗,” “social∗ robot∗,” “social∗ assistive robot∗,” “companion∗ robot∗,” “emot∗ robot∗,” “healthcare robot∗,” “robot∗ pet∗,” “home-care robot∗,” “assist∗ robot∗,” and “care robot∗.” Their associated MeSH terms were “robotics” and “artificial intelligence.” Free words used for the outcome included “accepta∗” and “attitude∗.” The use of the asterisk (∗) enables the word to be treated as a prefix. Screening of the abstracts and later the whole article was done by two authors.

### 2.3. Inclusion and Exclusion Criteria

To be included in this review, articles had to be written in English and showing initial results (qualitative or quantitative empirical data) related to acceptance of SARs (or to be used) by elderly users. Moreover, the articles had to be focused on use of SARs to support independent functioning and improved safety at home or in similar environments.

The exclusion criteria were (i) studies of purely ancillary geriatric care robots, such as intelligent wheelchairs or exoskeleton walkers, and (ii) studies reporting human-robot interactions or user input and literature reviews. Two independent reviewers performed the study selection. The relevancy of an article had to be judged by both reviewers. In cases of disagreements between the two reviewers, the first author with experience in robot acceptance research was involved to reach a consensus.

### 2.4. Study Selection Process

Articles were screened using EndNote X9. Screening of abstracts and the whole article was done by two authors. The search strategy identified 1187 unique citations, among which, based on their titles and abstracts, 207 articles were considered to be potentially relevant (Figure 1). After full-text reviews, 35 papers were retrieved for full-text screening. In cases of ambiguity, selection and exclusion were discussed with the first author to achieve 100% consensus on study inclusion. Finally, the selection process resulted in 35 articles that were included in the review.

### 2.5. Data Extraction and Data Analysis

One of the authors analyzed the included articles, summarized the data, and listed the emerging themes. The other author did not interfere in reviewing the data and adjusted the summary topic by extending or merging the topics and subtitles. Finally, the two authors reached a consensus on identified themes and subthemes. Data charting and table preparation were performed using Microsoft Excel (2016 version). Data regarding the location and year of publication, the population under study, technology acceptance models, and measurements of SARs were obtained, charted, and subjected to thematic analyses.

## 3. Results

### 3.1. Description of the Included Studies

The selected articles had been published between 2006 and 2021, with 71.4% (*N* = 25) of the articles published between 2015 and 2021, whereas 28.6% (*N* = 10) were published between 2006 and 2015. The articles were developed from studies conducted in 14 countries, with most of them in the United States (5, 14.3%), China (5, 14.3%), Netherlands (5, 14.3%), France (3, 8.6%), and Germany (3, 8.6%).

Various methods were used to evaluate acceptance, with quantitative analysis (25, 71.4%) being the most commonly method. Fifteen of the included articles used quantitative descriptive methods, nine used quantitative nonrandomized methods, and only one was a randomized controlled trial (RCT). Furthermore, seven articles used mixed methods combining interviews or observations with a questionnaire or objective measurements (20%). Three of the articles used single quantitative (interviews or focus groups) methods to collect information. The studies were predominantly based on self-report questionnaires (37.1%, 13/35), such as the Godspeed questionnaire [18], and the negative attitudes toward robots' scale [19]. Characteristics of the included studies are shown in Table 1.

### 3.2. General Attitudes towards Using SARs

Sixteen studies presented results on acceptance of SARs, among which 12 studies reported a positive attitude acceptance of SARs, indicating a positive general attitude towards using these robots. It was also evident that even the elderly, who are not technologically advanced, have shown interest in the robotic platform and think they can properly control the robots [28]. In the study by Kodate et al., about 178 (77%) of respondents reported that they were open to the use of home-care robots [40]. The three other studies reported that older adults had negative attitudes towards the idea of SARs in aged care [15, 29, 47]. Furthermore, they showed low intentions to use the robot.

### 3.3. Technology Acceptance Theory Models

The retrieved studies showed the willingness of researchers to use the existing theories (15, 42.9%). Three explicit theoretical framework(s) were reported, including the Technology Acceptance Model (TAM) [24, 35, 39], UTAUT model [12, 18, 25, 34, 45], and Almere model [11, 14, 15, 37, 38, 43].

Most of the studies that relied on theoretical framework added constructs to capture the influence of context-related factors on acceptance. For instance, there was a hedonic or pleasure-oriented use of technology of SARs, which would help offer interaction possibilities to build long-term relationships with users. Chen et al. argued that it is essential to examine the role of entertainment-oriented uses of SARs by older people [24]. Such evaluation will elucidate on technology acceptance of SARs in older people [41]. According to Lehmann et al., technology acceptance was dealt with in different models. However, most of these models only focused on cognitive and social factors of technology acceptance, and little attention has been given to emotions of older adults towards SARs [42]. Robots that support everyday activities can trigger human emotions, such as “fear,” “emotional involvement,” and “potential threat.” Therefore, more attention should be given to the emotions of older people when interacting with robots because emotions and attitudes influence their responses [27].

### 3.4. Factors Associated with Technology Acceptance

We categorized the factors that affect the attitudes of the elderly toward SARs into three major themes: individual characteristics, assistive technology characteristics, and social factors. Individual characteristics include age, gender, educational background, and technical experience. Assistive technology characteristics include effectiveness, image appearance, and matching technical efficiency with user expectations while psychosocial factors include fear of use/anxiety, fear of becoming lonely/stigmatization, and influence of the family and community (Table 2).

### 3.5. Individual Characteristics

Demographic characteristics of the elderly were associated with technology acceptance of SARs. Age is one of the major epidemiological factors influencing technology acceptance. Younger people are more willing to accept SARs, compared to older people [15, 35]. The influence of gender on technology acceptance remains uncertain. However, women showed a more positive attitude towards SARs than men and had a significantly higher perception of the roles of robots in reminding about medications, meal times, and drinks [44]. Two studies reported insignificant differences in attitudes towards SARs, regardless of gender [20, 41]. Louie et al. [43] reported that older people with a high level of education were more willing to interact with robots, which could have been because educated older adults had better recognition of the ability of SARs. Another study reported comparable findings that older adults with high education and medical backgrounds have more positive attitudes toward SARs [38].

Technical experience reduces the anxiety of using robots, thereby increasing the perceived ease of using robots [49]. In addition, live demonstrations on the use of robots can clarify the functions and benefits of robots and promote the needs of SARs for the elderly [22, 43]. Extraversion has been associated with positive attitude changes toward close correlations of individuals with robotics (*r* = 0.619) and positive attitude changes toward psychological conditions (*r* = 0.581). In contrast, neuroticism was negatively correlated with robotics (*r* = −0.582) [27]. Specific personality traits might be indicators of attitude changes associated with specific domains of social interactions.

### 3.6. Concerns/Problems regarding Robots

Several studies have found that appearance designs of SARs are an important factor affecting their acceptance by elderly people [14, 22, 33, 41, 43, 45]. Lifelike expressions of robots, beautiful faces, and nonthreatening appearances are attractive. Moreover, anthropomorphic voices can also reduce the difficulty of understanding.

The match between technical performance and user expectations is another essential factor. The willingness of older people to use robots was directly impacted by whether the features of robots met the needs of the people. The actual effect of SARs affects the willingness of older adults to use robots [18, 31, 38, 41, 46, 48]. The elderly also emphasized the importance of risk prevention and healthcare applications, such as falls, safety detection of critical situations, and alarms when in danger [14]. Some elderly users reported that frequent failure of voice control and robot interactions reduced their willingness to use robots because they felt easily frustrated [15].

### 3.7. Social Factors

Elderly users of the technology felt that the robot would make them feel older, more fragile, and frail. The main challenge to robot acceptance in the elderly is associated with the stigma brought about by robots, as reported by Park et al. [50]. This could be because assistive technology is related to loneliness, dependence, disability, and aging among the elderly [14, 15]. Some older adults expressed worries that robots will weaken their living abilities and limit their connections with family members and thus opposed the use of robots [15, 48]. Moreover, the elderly were worried about leakage of their privacy in case they used SARs [15].

## 4. Discussion

The framework map scientific literature aims at evaluating the technology acceptance of SARs by the elderly in care contexts.

The first objective of this review was to synthesize the evidence base for acceptance of SARs in real-world elderly care. Although there have been marked advances towards answering this question, no definitive conclusions have been reached. Compared to the literature on artificial intelligence, studies on SARs acceptance among older adults are few. In this review, 35 studies met the set inclusion criteria, with most of them having been published after 2013 (80.0%). In the past two years, the number of publications has significantly increased (31.4%). A study that assessed the influence of social abilities of a robot on elderly users' attitudes towards and acceptance of robots in eldercare institutions was conducted by Heerink et al. and published in 2006 [34]. The newest similar work was published in 2021 by Harrington et al. [33], which was an action research for three years on older people in their own homes. Thus, assessment of acceptance of SARs technologies in elder care is an emerging study field.

We found significant differences in acceptance of SARs among most older adults, which could have been due to various reasons. First, attitudes toward robots differ among users who come from varied cultural backgrounds and live in various environments [51]. Due to different countries in which researchers are located, there may be variations in assessment tools due to varying cultural backgrounds and population characteristics [2]; therefore, the obtained information may be scattered. Second, the perception of SARs may also change over time (e.g., aging of end-users and changes in their health) [37] or during the use of SARs (due to increasing familiarization and developing dependence) [52].

Advances in technologies have initiated the development of suitable approaches to improve the acceptance of robot technologies among older adults. It has been documented that SARs are necessary for overcoming the technical challenges. Efforts (i.e., adjusting the designs of robots) have aimed at improving the acceptance of SARs by the elderly. Portugal et al. [53] suggested designing robots in a modular way (i.e., possible to change or extend their functionality if necessary), which can partially overcome the limitations of not accepting SARs due to functional challenges. Future features should be personalized to suit each user's health needs, such as smoke detection and reading aloud capabilities [32].

The second objective of this review was to summarize the applications of technology acceptance theory in SARs designs and research processes. In medical contexts, two models, such as technology acceptance model (TAM) and unified theory of acceptance and use of technology (UTAUT), were established to be the most pertinent and widely used technology acceptance models. Both TAM and UTAUT are oriented towards a wide range of technologies. The Almere model, whose foundation is based on a validated technology acceptance model (UTAUT), proposed an assisted social robot acceptance model specifically by Heerink [37]. Compared to TAM and UTAUT, the Almere model reflects the complex psychological states of elderly people when they accept a new technology. Furthermore, the strengths of the Almere model [11] are that it is a concise quantitative measurement (e.g., a 41-item Likert-type questionnaire).

The general idea of theoretical models is to test for correlations between all potentially influential factors and technology acceptance. These models can clearly show the relationship between variables and their direct or indirect effects on acceptance. Despite limitations to existing measurement frameworks, often, the theoretical models were bottom-up, data-driven approaches that list simple regression results, which lack overall grasp of characteristics of robotics and in-depth analyses of technology-related theories. The SARs had characteristics that distinguish them from other assistive technologies. The SARs entertain and help people in their everyday tasks in environments in which they live (home and recreational environments). They tend to be highly autonomous and can safely interact with untrained people in unstructured environments. Technology characteristics make it more challenging to encourage the acceptance of SARs. For instance, the Almere model is limited because it does not incorporate human factors, such as robot experience. Thus, the existing knowledge lacks a holistic view of robot acceptance, including people, robots, tasks, environments, time, and their interactions. Despite the significance of technology models with regard to acceptance, they should only be used as maps.

The third objective of this review aimed at identifying the currently used tools and approaches for assessing the acceptance of robots in elderly care. We established that there is a need for further reviews of technology acceptance assessment tools for SARs.

Most of the included articles involved quantitative data collection methods using various constructs and questionnaires. The acceptance of SARs was primarily assessed by constructing technology acceptance models to compile questionnaires [12, 14, 18, 22, 23, 25, 26, 29, 31, 37, 40, 42, 45, 47]. Furthermore, self-developed questionnaires were also used [19, 20, 27, 41, 43, 46]. There were considerable variations between the reliability and validity of other research instruments, making it difficult for future researchers to replicate the studies and compare the results of different studies to identify trends and commonalities.

Measurement of the acceptance of robots using self-report questionnaires is relatively simple because it provides a direct and subjective response to the user's opinion. It allows the researcher to have a rough idea of the user's attitudes towards the robot, which is useful when determining the suitability of a particular intervention for a client. However, there are no objective indicators for evaluating user acceptance, which is insufficient to accurately and effectively assess user acceptance levels. Therefore, future studies should use multiple methods to assess technology acceptance because combining self-reported data with recorded data to obtain more objective data is possible. For instance, a combination of individual and group interviews with older adults as well as direct observations and recording of the use of robot technologies at home would help in accurate and reliable assessment of technology acceptance.

There is a need to consider the timing and context of assessing the acceptance of robot technologies. The studies in this review assessed technology acceptance without reference to factors related to contact time. It is clear that people's first impressions of SARs are often positive. However, preferences and attitudes of users may drastically change, especially in the case of the elderly in their homes [54]. These impressions are valuable for human-robot interaction scenarios. Due to the late development of SARs in China, a limited number of studies have been conducted on long-term use and benefits of SARs in domestic conditions. Therefore, studies should be conducted in private homes and over more extended periods to explore the various factors that change over time.

Our findings also revealed various barriers and facilitators of SARs acceptance. The difficulties and challenges in SARs research might be attributed to individual characteristics, concerns/problems regarding robots, and social factors.

The acceptance of new technologies by older people is complex. Several factors influence the acceptance of SARs by elderly individuals. Most of these factors are associated with performance expectations of the technology. For example, older people attach great importance to safety issues [14, 22] and perceived risks [48]. The need for SARs by older people was based on their health conditions, which should be considered in future research. Emotional companionship has also been reported to be an essential factor influencing robot acceptance [38, 41]. Some participants raised ethical concerns [15, 48]. In addition, the community has marked influences on willingness to use the technology by older people.

The factors affecting the acceptance of SARs by older people are complex. Thus, practical designs and implementation principles of robotic technologies should be based on the factors found in literature. Moreover, there is a need for further studies to clarify which factors are most important in influencing technology acceptance of SARs. These studies will inform on designs of SARs to relieve the pressure of aging populations.

## 5. Limitations

This review had some limitations. First, there may have been gray literature not included in this review because the SARs in elder care are an emerging science. Therefore, review findings may not have fully reflected technology acceptance of robotics.

Second, findings on technology acceptance in the current review were limited by how technology acceptance data were collected. Sixteen of the 35 studies used a single, structured approach (through structured questionnaires or reports generated by the technology). Therefore, this approach would have restricted the study investigators from identifying novel or unexpected findings related to acceptance of robots.

## 6. Conclusions

Research on technology acceptance of SARs is still in the developmental stages. The current theoretical models and measurements do not address the comprehensive and in-depth understanding of SARs technology acceptance by the elderly. The impact factor of technology acceptance might be correlated with individual characteristics, concerns/problems regarding robots, and social factors. Thus, further research should be conducted to explore a generic and specific framework to identify technologic acceptance of SARs. This review leaves the stage open for researchers to provide some insights and helpful information for future research into the designs of SARs. The technology acceptance theory can be informed by exploring the current extending models and boundary conditions. This review also provides guidelines to help designers to better adapt robotic innovations from a practical point of view in the care sector to benefit older adults and increase the chances of robot-supported independent aging.

## Figures and Tables

**Figure 1:** Article selection process.

**Table 1:** Study types, participants' characteristics, acceptance measurement, and study designs.

Article	Time	Country	Study design	Acceptance measurement	Population	Participants
Baisch et al. [20]	2017	Germany	Quantitative descriptive	Robot acceptance questionnaire	Old adults	29

Bajones et al. [19]	2019	Austria, Greece, Sweden	Quantitative descriptive	Negative attitudes toward robots scale (NARS)	Old adults	16

Beer et al. [21]	2017	United States	Quantitative nonrandomized	Robot opinions; assistance preference checklist	Old adults	12

Cavallo et al. [22]	2018	Italy	Quantitative nonrandomized	Self-report questionnaires	Old adults	45

Chen and Lou [23]	2020	China (Hong Kong)	Randomized control trials	Questionnaire of senior technology acceptance model (S-STAM)	Old adults	103

Chen [12]	2018	China	Quantitative descriptive	The UTAUT questionnaire	Old adults	277

Chen et al. [24]	2017	United States	Mixed	Robot opinions questionnaire	Old adults	16

Chien et al. [25]	2020	China (Taiwan)	Quantitative nonrandomized	Self-report questionnaires	Older adults/younger	80

Chiu et al. [26]	2021	China (Taiwan)	Quantitative descriptive	Self-report questionnaires	Middle-aged and older adults	273

Damholdt et al. [27]	2015	Denmark	Quantitative nonrandomized	Attitudes toward social robots scale (ASOR-5)	Old adults	14

D'Onofrio et al. [28]	2019	Italy and Japan	Qualitative	Interview outline	Old adults/health care workers	17/36

Dudek et al. [29]	2020	Germany	Quantitative descriptive	Self-report questionnaires	Old adults	28

Esposito et al. [30]	2020	Italy	Quantitative nonrandomized	Robot acceptance questionnaire (inside the H2020 project empathic)	Old adults	90

Ezer et al. [31]	2009	United States	Quantitative nonrandomized	Self-report questionnaires	Older adults/younger	117/60

Gasteiger et al. [32]	2021	New Zealand	Qualitative	Interview outline	Old adults	6

Harrington et al. [33]	2021	United States	Quantitative descriptive	The perceptions of social robots questionnaire	Old adults	51

Heerink et al. [34]	2006	Netherlands	Mixed	The UTAUT questionnaire	Old adults	40

Heerink et al. [35]	2008	Netherlands	Quantitative descriptive	Self-report questionnaires	Old adults	70

Heerink et al. [36]	2009	Netherlands	Quantitative descriptive	Self-report questionnaires	Old adults	40

Heerink et al. [11]	2010	Netherlands	Quantitative descriptive	The Almere questionnaire	Old adults	188

Heerink [37]	2011	Switzerland	Quantitative descriptive	The Almere questionnaire	Old adults	66

T. Huang and C. Huang [38]	2019	China (Taiwan)	Mixed	Self-report questionnaires	Old adults	148

Klamer and Allouch [39]	2010	Germany	Qualitative	Interview outline	Old adults	3

Kodate et al. [40]	2020	Ireland	Quantitative nonrandomized	Self-report questionnaires	Old adults/family care/health care workers	114/8/56

Kuo et al. [41]	2009	New Zealand	Quantitative nonrandomized	Attitudes toward healthcare robots scale (ATHR); robot attitudes scale (RAS)	Old adults/adults	57

Lehmann et al. [42]	2021	Switzerland	Quantitative descriptive	Self-report questionnaires	Old adults	142

Louie et al. [43]	2014	Canada	Quantitative descriptive	Robot acceptance questionnaire	Old adults	46

Łukasik et al. [44]	2021	Poland	Quantitative descriptive	Users' needs questionnaire	Old adults	166

Pino et al. [14]	2015	France	Mixed	Self-report questionnaires	Old adults	25

Piasek and Wieczorowska-Tobis [18]	2018	Poland	Quantitative descriptive	The godspeed questionnaire; the Almere questionnaire	Old adults	5

Sinnema and Alimardani [45]	2019	Netherlands	Quantitative nonrandomized	The UTAUT questionnaire	Older adults/younger	52/13

Smarr et al. [46]	2013	United States	Mixed	Robot opinion questionnaire	Old adults	21

Takanokura et al. [47]	2020	Japan	Quantitative descriptive	Self-report questionnaires	Elderly users/healthcare workers	63/4

Wu et al. [15]	2014	France	Mixed	Robot acceptance questionnaire	Old adults	11

Ziefle and Valdez [48]	2015	France	Mixed	Self-report questionnaires	Old adults	25

**Table 2:** Factors affecting the acceptance of SARs.

Theme	Factor	Ref
Demographics	Age	21, 40, 42, 46, 48
	Gender	18, 21, 40, 42
	Technical interest	15, 38, 44
	Previous technological experience	12, 14, 21, 30, 37, 42, 45, 48
	Physical environment and conditions	14, 15, 23, 37, 38, 46, 48
	Education background	21, 34, 37, 42

Concerns/problems regarding technology	Technical issues (simple function, control not well, limited conversation abilities, high maintenance)	11, 14, 15, 21, 33, 35, 38, 48
	Meet needs (entertainment, emotional support, improve the quality of life, increased safety, companionship, increased independency, increase communication and social life)	14, 15, 18, 21, 23, 33, 37, 40, 43, 44, 46
	Robot appearance	14, 15, 21, 32, 38, 42,

Psychosocial factors	Fear of use/anxiety	42, 44, 45, 48
	Influence of family and community	30, 32, 37
	Fear of becoming dependent/lonely	15, 18, 44
	Fear of revealing privacy	15
	Feeling of stigmatization	15, 48

## Data Availability

The data used to support the findings of this study are included within the article.
